# Diagnosis of Heterotopic Pregnancy Using Ultrasound and Magnetic Resonance Imaging in the First Trimester of Pregnancy: A Case Report

**DOI:** 10.1155/2012/317592

**Published:** 2012-12-04

**Authors:** Sue Yazaki Sun, Edward Araujo Júnior, Julio Elito Júnior, Liliam Cristine Rolo, Felipe Favorette Campanharo, Stéphanno Gomes Pereira Sarmento, Luciano Marcondes Machado Nardozza, Antonio Fernandes Moron

**Affiliations:** Department of Obstetrics, Federal University of São Paulo (UNIFESP), 05303-000 São Paulo, SP, Brazil

## Abstract

Heterotopic pregnancy is a condition characterized by implantation of one or more viable embryos into the uterine cavity while another one is implanted ectopically, particularly into the uterine tube. Its occurrence has increased drastically over the last few years due to assisted reproduction procedures. In general, the diagnosis is made during the first trimester by using endovaginal two-dimensional ultrasound (2DUS), through observing a complex para- or retrouterine mass in association with a viable uterine pregnancy. However, under some conditions such as atypical ultrasonographic presentations, 2DUS does not clarify the situation whereas magnetic resonance imaging (MRI) of the pelvis is able to do so. We present the case of a pregnant woman in her fifth pregnancy, with a clinical condition of lower abdominal pain and pallor. Endovaginal 2DUS showed a complex voluminous mass in the left pelvic region in association with a viable intrauterine pregnancy. 2DUS in power Doppler mode showed “ring” vascularization, compatible with an ectopic gestational sac. MRI was of great importance in that it suggested that the mass had hematic content, which together with the clinical features, indicated that laparotomy should be performed. This surgical choice was essential for the woman to achieve a clinical improvement and for good continuation of the intrauterine pregnancy.

## 1. Introduction

Heterotopic pregnancy is defined as the presence of simultaneous pregnancies in two different implantation sites. The most frequently observed manifestation is the presence of an intrauterine pregnancy and an ectopic pregnancy that is usually located in the uterine tube, most commonly in its ampullary portion (80%) [1]. The incidence of heterotopic pregnancy is around 1/30,000 in spontaneous pregnancies. Among pregnancies resulting from assisted reproduction techniques, the incidence is greater, ranging from 1/100 to 1/3,600 [2, 3]. Diagnosing this clinical occurrence is a challenge, given the complexity of the possible clinical and laboratory manifestations. 

We present a case of heterotopic pregnancy during the first trimester that was diagnosed by using two-dimensional ultrasound (2DUS) and magnetic resonance imaging (MRI).

## 2. Case Presentation

A 33-year-old pregnant woman in her fifth pregnancy (one cesarean and two previous premature abortions, with right-side salpingectomy due to an ectopic tubal pregnancy) was referred to the Department of Obstetrics of the Federal University of São Paulo (UNIFESP) during her 12th week of pregnancy. She had a complaint of intermittent hypogastric pain that partially improved with ordinary analgesics, accompanied by mucocutaneous pallor, dysuria, and rectal tenesmus. 

The pregnant woman had initially been hospitalized for five days at another service, where she received transfusion of three red blood cell concentrates due to anemia (Hb: 6.8 mg/dL). Endovaginal 2DUS was performed using the Voluson E8 device (General Electric Healthcare, Zipf, Austria) with the RIC 5-9 transducer, from which a normal pregnancy of 10 weeks and 4 days was diagnosed, along with presence of a heterogeneous irregular mass in the left abdominal pelvic region, with dimensions of 12.8 × 11 × 10 cm (volume: 745 mL). This mass presented “ring” vascularization on power Doppler, indicative of a gestational sac (Figure 1). The ovaries were characterized as juxtaposed with the above formation and presented the usual dimensions and texture. The woman had made use of emergency contraception.

On hospitalization in our service, she was pale, with blood pressure of 120 × 70 mmHg and heart rate of 104 bpm. Her abdomen was tense and she presented a palpable mass extending down to 6 cm above the pubic symphysis, which was painful on palpation, without signs of peritoneal irritation. 

The posterior vaginal fornix presented bulging that was painful upon touching, with Hb of 8.4 mg/dL. To complement and clarify the diagnosis, MRI of the pelvis was performed using a Sonata Maestro Class 1.5 T device (Siemens, Erlangen, Germany) with 8-channel dedicated coils. The MRI was performed using the turbo spin echo (TSE) technique, gradient echo (FLASH), and T1 and T2-weighting, from which axial and coronal images were obtained. A large left adnexal mass that probably had red blood cell content was observed, which measured 13 cm along its greatest diameter (Figure 2).

In view of the unstable clinical features, it was decided to perform exploratory laparotomy. This showed the presence of a red blood cell accumulation at an advanced organizational stage, obliterating the bottom of the pouch of Douglas. A volume of 500 mL of coagulum came out from the left adnexa (Figure 3(a)). Left salpingooophorectomy was performed, and the resultant anatomopathological examination was conclusive for trophoblastic tissue (Figure 3(b)). The pregnant woman evolved with improvement of her clinical condition and is currently undergoing prenatal followup, using progesterone, without complications at the present moment.

## 3. Discussion

Because of the high risk of tubal rupture, the importance of early diagnosis and treatment for the ectopic pregnancy becomes clear in the light of this paper. Around 50% of heterotopic pregnancies are asymptomatic [4]. When symptomatic, the main clinical manifestations are abdominal pain due to peritoneal irritation, adnexal mass with or without vaginal bleeding and hypovolemic shock. Fortunately, in this case, the classical symptoms of ectopic pregnancy were present to guide the clinical diagnosis. However, clinical manifestations are more frequent in situations of tubal rupture.

To assist in early screening and diagnosing of ectopic and heterotopic pregnancies, *β*-hCG serum assaying, along with vaginal 2DUS, can be routinely used in prenatal examinations during the early stages of pregnancy. However, heterotopic pregnancies may be obscured in the presence of intrauterine pregnancies, due to the difficulty of differential diagnosis between ectopic pregnancy and hemorrhagic corpus luteum, abortion, neoplasia and adnexal torsion. Many of these can be associated with normal pregnancies, thus resulting in delayed diagnosis [5].

In normal pregnancies with blood *β*-hCG levels above 1,500–2,000 mIU/mL, the intrauterine image of the pregnancy should already be detectable. However, identifying the intrauterine image does not exclude the possibility of heterotopic pregnancy, which is more frequent with fertility treatments [2, 3]. Thus, adequate viewing of the adnexa becomes necessary in all assessments on the start of pregnancy. 

The most commonly present extrauterine images in transvaginal 2DUS in heterotopic pregnancies consist of complex cysts or adnexal masses, which may comprise hematosalpinx, tubal ring, or even a live embryo, with or without accompanying free fluid in the peritoneal cavity [6]. However, 2DUS may often be indeterminate, and in such cases, MRI of the pelvis may be used to assist in the diagnosis [7], as shown in the present paper. Structures located in the adnexal region that are similar to the gestational sac, or even cystic formations, may be identified on MRI. Occasionally, it is possible to observe a thickened tubal wall with cystic content within, or even the presence of hematomas due to the tubal rupture (low T2 signal intensity) [7]. In the present case, MRI was important for indicating treatment via laparotomy, since 2DUS was not able to clarify whether heterotopic pregnancy was present.

Thus, if adnexal changes are suspected in an ongoing pregnancy, especially in pregnancies resulting from infertility treatment, both 2DUS and MRI are important in making the differential diagnosis of heterotopic pregnancies.

In summary, we presented a case of heterotopic pregnancy in which MRI was essential to complement the diagnosis, thereby allowing adequate surgical treatment, which enabled evolution of the intrauterine pregnancy. Because of the rarity of heterotopic pregnancy, we recommend that MRI of the pelvis should be used in cases of initial pregnancy associated with retrouterine or parauterine masses diagnosed by means of 2DUS.

## Figures and Tables

**Figure 1:** (a) B-mode endovaginal 2DUS showing a large irregular heterogeneous mass in the left pelvic abdominal region; (b) endovaginal 2DUS in power Doppler mode showing “ring” vascularization, indicative of a gestational sac. 2DUS: two-dimensional ultrasound.

**Figure 2:** (a) T2-weighted sagittal sequence MRI, showing uterus with 12-week conception in the anterior region and a complex mass occupying the retrouterine region; (b) adnexal T2-weighted sequence MRI, showing large cystic mass with “onionskin” appearance, which might correspond to multiple episodes of organized bleeding. MRI: magnetic resonance imaging.

**Figure 3:** (a) Intraoperative situation, showing the presence of a great amount of coagulum in the pelvic cavity as well as lesions in the left uterine tube and ovary; (b) surgical specimen, showing left ovary with intact corpus luteum and small fragment of the left uterine tube.
